# Bolus Feeding Via Gastric Versus Oral Routes in Very Preterm Neonates

**DOI:** 10.34763/jmotherandchild.20242801.d-23-00060

**Published:** 2024-02-27

**Authors:** Rita P. Verma, Deepank Sahni, Joshua Fogel

**Affiliations:** Nassau University Medical Center, East Meadow, NY 11554, NYC Health+ Hospitals/South Brooklyn Hospital, Coney Island, NY 11235; Nassau University Medical Center, East Meadow, New York, 11554; Nassau University Medical Center, New York, NY 11210

**Keywords:** Very preterm neonates, Bolus orogastric feeding, Enteral nutrition, Postnatal Catch-up growth, Duration of hospitalization

## Abstract

**Background:**

We intend to investigate the association of bolus orogastric tube (BOG) and nipple bottle (N) feedings with postnatal growth in very premature neonates (VPN: gestational age between 28 and 33 weeks).

**Material and methods:**

The days of life (DOL) to achieve full combined oral and gastric enteral nutrition (FEN) and attain body weight (BW) of 2200 g (Wt22) and the length of hospitalization (LOH) were retrospectively associated with clinical and BOG and N feeding-related variables via multivariate regression analyses. Correlations were performed to ascertain the strength of associations.

**Results:**

In a cohort of 127 VPN, FEN demonstrated negative associations with gestational age (GA) and LOH and Wt22 with birth weight (BW). FEN showed positive associations with nil by mouth and intravenous fluid-nutrition days and with DOL to start and achieve full nipple feeding. LOH was associated with days on antibiotics and DOL to start and achieve full nipple feeding. Wt22 was associated with DOL to achieve full nipple feeding. The start day of BOG feeding had no independent associations and weak, highly significant positive correlations with Wt22, LOH, and FEN.

**Conclusion:**

Bolus orogastric tube feeding has no independent implications for postnatal growth, duration of hospitalization, or chronological age to attain full enteral nutrition in VPN unless combined with nipple feeding to provide enteral nutrition. Oral bottle feeding accelerates postnatal catch-up growth and full enteral nutrition acquisition while reducing hospitalization duration. Initiating nipple feeding at 32 weeks of postmenstrual age may be safe in stable VPN. Antibiotic therapy increases hospitalization duration.

## Introduction

Nipple feeding via bottle in preterm neonates is provided by contingent care based on readiness cues. Acquisition of this developmental function is governed by neurological maturation and autonomic, motor and behavioral state organization [1]. Feeding behavior in preterm infants matures between 33 and 36 weeks after conception, and sucking-swallowing coordination is well developed by 34–36 weeks of gestation [2,3,4,5].

The requirement of nutrients that would match the in-utero accretion rate is significantly high during the postnatal period in preterm infants [6]. The physiological rate of weight gain in these infants is about twice as much as their term counterparts [7]. Clinical decisions regarding the type, volume, osmolality and rate of advancements of enteral feeding play critical roles in their postnatal growth [8,9]. According to a recent report, 22–25% of the neonatal intensive care unit (NICU) population comprises neonates born between 28 and 33 weeks [10]. Infants in this group, categorized as very premature neonates (VPN), are deprived of the nutritional accretion and rapid weight gain acquired during the 3^rd^ trimester of intrauterine life.

Enteral nutrition is provided via gastric tube as a continuous drip or intermittent bolus in preterm neonates until they are clinically ready for bottle feeding [9, 11, 12]. Studies that reported the benefits of early trophic gastric tube feeding on postnatal growth and development did not separate continuous and bolus gastric feeding practices. These results were not supported in a Cochrane review [13].

We investigated the associations of postnatal days taken to achieve full enteral feeding (FEN), to gain the minimum body weight consistent with term status, and the duration of hospitalization with enteral nutrition provided by intermittent bolus through an orogastric tube (BOG) and orally with nipple and bottle (N) in VPN. The aim was to examine the effects of bolus feedings given via gastric and oral routes on postnatal growth.

## Material and methods

This retrospective cohort single-center study was conducted at a suburban teaching hospital in Long Island, New York. All preterm infants born between 27,0/7 and 32,6/7 weeks of gestational age (GA) admitted to the NICU during a designated period were candidates for the study. Those who suffered from congenital anomalies of the gastrointestinal, respiratory, genitourinary, cardiovascular, central nervous, intrauterine growth, skin, and other organ systems or expired during the study period were excluded. The following neonatal variables were studied in the enrolled infants: GA; birth weight (BW); gender; mode of delivery (cesarean or vaginal); ethnicity; Apgar scores at five minutes of life; the receipt of any respiratory support including oxygen (O_2_), distending pressure or mechanical ventilation; necrotizing enterocolitis in stage two or over (NEC); patent ductus arteriosus (PDA) as diagnosed via echocardiography of any size; the total number of days on antibiotics as administered for suspected, clinical or culture-proven sepsis; and the length of hospitalization (LOH). The caretaking team made all clinical decisions and followed the standard sepsis evaluation and treatment protocols as per American Academy of Pediatrics guidelines. The variables related to neonatal nutrition were as follows: day of life (DOL) when enteral feed was started by nipple (N) or as bolus via OG tube (BOG); DOL and GA when nipple feeding was started; the total number of days on parenteral fluids including 10% dextrose solution or hyperalimentation; use of any volume of colostrum and expressed maternal breast milk; DOL to reach full enteral feeding by OG tube, nipple or both combined (FEN); DOL of achieving full enteral feeding via nipple; the total number of days when the infant was nil by mouth (NPO); daily weight gain; and the number of days to achieve a bodyweight of 2200g (Wt22). Expressed maternal breast milk for the first five post-delivery days was considered as colostrum. The following maternal variables were included in the study: hypertension or diabetes mellitus of any severity during pregnancy and any receipt of steroids, magnesium sulfate, or antibiotics within four weeks of delivery. The neonatal and maternal variables were analyzed for their association with LOH (days), FEN (days), and Wt22 (days) as the outcome variables. The body weight of 2200 g was selected as it is the tenth percentile for 37 weeks of gestation, which defines term status. The GA was determined by the last menstrual period dating and fetal ultrasound and was confirmed at birth by incorporating the standard Ballard scoring in the physical examination.

The neonates were started on intermittent bolus trophic feeds via OG tube with 10–20 ml/kg/d of expressed colostrum, maternal breast milk (MBM) as available, and mixed with the premature Enfamil 20 calories (PE20) formula during DOL 0–3 as allowed by the clinical stability [13]. Standard soft polyvinyl chloride or silicone feeding tubes of appropriate size (NeoMed Enfit) were used. OG tube was removed, and a new one was inserted for each feeding. Infants were started on parenteral nutrition within the first 24 hours of life with 10% dextrose solution, 2–3 g/kg/d of amino acids, and 1–2 g/kg/d of lipids and gradually increased to a maximum of 4 g/kg/d of protein and 3 g/kg/d of lipids while adjusting for the enteral nutrition. Initial fluids were provided at 80 ml/kg/day The volume of the feeding aliquot was advanced after being on trophic feeds for 3–7 days, as per feeding tolerance and clinical condition, by a maximum of 20–30 ml/kg/day to reach the total volume of 140–150 ml/kg/day and 110–120 calories/kg/day, which were considered as full feeds.

Bottle nipple feeding was tried at approximately 32–33 weeks of postmenstrual age by following the neonatal cues for readiness, such as synchronous vigorous nonnutritive sucking without bradycardia, oxygen desaturation, or apnea. Initially, nipple feeding was tried every 8–12 hours with full or partial aliquot as tolerated without significant change in vital signs or clinical status. The nipple feeding was interrupted, and an OG tube was inserted for the remaining volume if the infant stopped nippling or the clinical status did not permit its continuation. The nipple feeding tolerance varied among infants and was clinically dealt with as needed. The recorded day of starting nipple feeding was not changed for analysis, even if it was interrupted for over 24 hours for any reason. The babies were not restricted from putting on the breast, but it was infrequent and was followed by bottle feedings as the major source of nutrition. Colostrum and expressed maternal breast milk were used as available. MBM was fortified to 22 calories per ounce when infants tolerated 40–60 ml/kg/d of enteral feeding and then to 24 calories per ounce. Premature Enfamil 24-calorie formula was introduced after 5–7 days of PE20 intake. Parenteral nutrition was supplemented and adjusted to the total volume of enteral nutrition. The Institutional Review Board approved the study before commencement.

## Statistical analysis

The numerical variables were analyzed as mean and standard deviation and the categorical ones as frequency and percentage. Skewed variables with zero values had one added to be logarithmically transformed. Univariate linear regression was conducted for each of the outcome variables. The multivariate linear regression with Beta co-efficient analysis included statistically significant predictors in the univariate analysis. Pearson correlation coefficient tests were utilized to estimate the strength of the relationship between variables. IBM SPSS Statistics Version 25 was used for all analyses. All *p*-values were two-tailed.

## Results

The clinical characteristics of the infants and mothers and the feeding-related neonatal variables are presented in Table 1. One hundred and thirty-four neonates were born during the study period, out of which seven were excluded for incomplete data and congenital anomalies. One hundred and twenty-seven eligible infants were included in the final analysis. Fifty-one percent of the infants were male, and 66.1% were non-Caucasian. The mean (standard deviation) of GA in infants was 30.6(1.9) weeks, and that of BW was 1482 (43.9) g. The mean (standard deviation) of FEN and that of Wt22 were 18.8(12.3) and 36.1(17.8) days, respectively, while that of the LOH was 44.8 (20.7) days.

**Table 1.** Maternal and neonatal clinical characteristics. (Data presented as mean (SD) for numerical and number (%) for categorical variables).

**Variables**	***n* = 127**
Gestational age (weeks)	30.6 (1.9)
Birthweight (grams)	1,482 (43.9)
Male	65 (51.2)
Non-Caucasian	84 (66.1)
Apgar at five minutes of life	7.8 (1.2)
Total number of days on antibiotics	5.2 (4.8)
Oxygen or positive pressure therapy	102 (80.3)
PDA	18 (14.2)
NEC	2 (1.6)
Maternal hypertension	43 (34.5)
Maternal diabetes mellitus	14 (10.9)
Antenatal steroids	117 (92.1)
Antenatal magnesium sulfate	108 (85.7)
Antenatal antibiotics	74 (64.2)
NPO days	4.7 (4.2)
Total days on intravenous fluids-nutrition	18.1 (13.49)
DOL when any feeding was started	3.4 (1.97)
DOL when gastric bolus feeding was started	3.6 (2.18)
DOL when nipple feeding was started	14.2 (14.52)
GA, when nipple feeding was started	32.4 (1.18)
DOL when full nipple feeding was achieved	25.7 (18.96)
Colostrum intake	80 (62.9)
Maternal breast milk intake	93 (73.2)
Daily weight gain	22.6 (6.85)
Length of hospitalization (days) (LOH)	44.8 (20.7)
Days to reach 2200 grams of body weight (Wt22)	36.1 (17.8)
Day of life when full feeding achieved (gastric and nipple feeding combined) (FEN)	18.8 (12.3)

NPO = nil by mouth, DOL = day of life, GA = gestational age (weeks), OG = orogastric tube.

Tables 2–4 present the linear regression analyses with values of unstandardized beta (B), standard error (SE), and probability (p) for FEN, LOH and Wt22. For all three outcome variables, several associations noted in the univariate analysis lost significance in the multivariate analyses. FEN had a negative association with GA and positive associations with NPO days, total days on intravenous fluid nutrition and DOL of starting and achieving full nipple feeding in the multivariate analysis (Table 2). LOH had a negative association with BW and positive associations with days on antibiotics and DOL of starting and achieving full nipple feeding (Table 3). Wt22 showed a negative association with BW and a positive association with DOL of achieving full nipple feeding (Table 4). Colostrum was associated with all three outcome variables in univariate but not multivariate analysis, while MBM was associated with LOH in univariate analysis only. The antenatal exposure to steroids did not show any associations in the regression analyses of any outcome variables at unstandardized beta (standard error) of 1.88(7.66) for LOH, 2.06(6.91) for W22, and −.27(4.93) for FEN in univariate analysis. Likewise, expressed in beta (SE), maternal hypertension −6.39(4.22) for LOH, −0.36(3.85) for Wt22, −5.03(2.71) for FEN], antenatal magnesium sulfate [6.46(5.76) for LOH, 10.36(5.13) for Wt22, 5.84(3.69) for FEN] and antenatal antibiotics [2.32(4.17) for LOH, −0.23(3.77) for Wt22, 0.75(2.69) for FEN] did not demonstrate significant associations in univariate analysis. Maternal diabetes mellitus had significant associations with LOH [−15(6.33), *p* < 0.05], Wt22 [−16.7(5.65), *p* < 0.001] and FEN [−8.59(4.11), *p* < 0.05] in univariate analysis which declined in the multivariate analyses. The strongest correlations were noted between DOL of achieving full nipple feeding and the LOH (*r* = 0.88 *p* < 0.001), Wt22 (*r* = 0.86, *p* < 0.001), FEN (*r* = 0.84, *p* < 0.001) and DOL of starting nipple feeding (*r* = 0.84, *p* < 0.001) (Table 5). DOL of starting nipple feeding also had strong correlations with Wt22 (*r* = 0.81, *p* < 0.001), LOH (*r* = 0.88, *p* < 0.001) and FEN (*r* = 0.83 *p* < 0.001). In contrast, DOL, when gavage feed was started, had weak correlations with LOS (*r* = 0.36, *p* < 0.001), Wt22 (*r* = 0.37, *p* ≤ 0.001), FEN (*r* = 0.4, *p* < 0.001) and DOL of starting nipple feeding (*r* = 0.38, *p* < 0.001). FEN correlated strongly with Wt22 (*r* = 0.8, *p* < 0.001), and LOH (*r* = 0.83, *P* < 0.001).

**Table 2.** Associations between clinical and nutrition supplementation variables with DOL to achieve full enteral feeding (FEN) via linear regression analysis.

**Variable**	**Univariate B (SE)**	**Multivariate B (SE)**
Gestational age (weeks)	−5.39 (0.33)^***^	−1.06 (0.52)^*^
Birthweight (g)	−0.03 (0.002)^***^	<0.001 (0.002)
Male gender	0.92 (2.47)	–
Non-Caucasian ethnicity	−0.85 (2.60)	–
Apgar score at five minutes of life	−4.45 (0.90) ^***^	0.24 (0.45)
Days on antibiotics	22.53 (3.05) ^***^	1.87 (1.95)
Oxygen or positive pressure therapy	15.52 (3.44) ^***^	−3.45 (1.89)
PDA	14.81 (3.47) ^***^	1.44 (1.78)
NPO days	15.12 (1.94) ^***^	4.30 (1.23)^**^
Colostrum intake	6.66 (2.63) ^***^	−1.63 (1.17)
Maternal breast milk intake	4.98 (2.91)	
Total days on intravenous fluid-nutrition	35.48 (1.90)^***^	14.48 (2.97)^***^
DOL when gastric bolus feed started	2.60 (0.52)^***^	0.29 (0.36)
DOL when nipple feeding started	0.81 (0.05)^***^	0.22 (0.07)^**^
GA, when nipple feeding was started	−0.57 (1.05)	–
DOL of achieving full nipple feeding	0.62 (0.04)^***^	0.14 (0.06)^*^
Daily weight gain (grams)	−3.73 (10.31)	–
Intercept	–	27.29 (17.52)

B = unstandardized beta, SE = standard error, Adjusted *R* square = 0.85.

* *p* < 0.05,

*** *p* < 0.001

NPO = nil by mouth, DOL = day of life, GA = gestational age (weeks)

**Table 3.** Associations between clinical and nutrition supplementation variables and the length of hospitalization (LOH) via linear regression analysis.

**Variable**	**Univariate B (SE)**	**Multivariate B (SE)**
Gestational age (weeks)	−8.84 (0.55)^***^	−0.87 (0.77)
Birthweight (g)	−0.04 (0.003)^***^	−0.02 (0.003)^***^
Male gender	3.27 (3.69)	–
Non-Caucasian ethnicity	3.92 (3.89)	–
Apgar at five minutes of life	−4.99 (1.47)^**^	1.10 (0.67)
Days on antibiotics	32.39 (4.92)^***^	6.57 (2.89)^*^
Oxygen or positive pressure therapy	24.99 (5.31) ^***^	−0.3 (2.65)
PDA	23.87 (5.36) ^***^	−0.68 (2.51)
Colostrum intake	12.26 (4.04) ^***^	1.29 (1.90)
Maternal breast milk intake	8.90 (4.50) ^*^	−0.87 (2.04)
NPO days	38.67 (5.17)^***^	1.07 (3.89)
Total days on intravenous fluid-nutrition	48.63 (3.54)^***^	5.08 (4.44)
DOL gastric bolus feed started	3.25 (0.81)^***^	−0.33 (0.52)
DOL when nipple feeding was started	1.37 (0.08)^***^	0.29 (0.12)^*^
GA when nipple feeding was started	−0.39 (1.57)	–
DOL when full nipple feeding achieved	1.05 (0.05)^***^	0.38 (0.10)^***^
Daily weight gain (g)	16.09 (15.25)	–
Intercept	–	60.07 (26.35)^*^

B = unstandardized beta, SE = standard error, Adjusted *R* square = 0.87, NPO = nil by mouth, DOL = day of life, GA = gestational age.

* *p* < 0.05,

** *p* < 0.01,

*** *p* < 0.001

**Table 4.** Associations between clinical and nutrition supplementation variables with number of days to reach 2,200 g (Wt22) via linear regression analysis.

**Variable**	**Univariate B (SE)**	**Multivariate B (SE)**
Gestational age	−7.28 (0. 15)^**^	−0.13 (0.49)
Birthweight (g)	−0.04 (0.001)^***^	−0.03 (0.002)^***^
Male gender	1.08 (3.18)	–
Non-Caucasian ethnicity	0.94 (3.36)	–
Apgar score at five minutes of life	−4.84 (1.25)^***^	−0.34 (0.43)
Days on antibiotics	22.24 (4.48) ^***^	1.26 (1.83)
Oxygen or positive pressure therapy	21.89 (4.81)^***^	−0.36 (1.89)
PDA	22.10 (4.81)^***^	0.24 (1.77)
NPO days	12.54 (2.88)^***^	1.98 (1.15)
Colostrum intake	10.80 (3.65) ^***^	0.25 (1.16)
Maternal breast milk intake	7.59 (4.06)	–
Total days on intravenous fluid-nutrition	40.84 (3.14)^***^	2.69 (2.81)
DOL when OG bolus feed was started	2.88 (0.69)^***^	0.37 (0.33)
DOL when nipple feeding started	1.12 (0.07)^***^	0.07 (0.08)
GA, when nipple feeding was started	−0.47 (1.35)	–
DOL of achieving full nipple feeding	0.87 (0.05)^***^	0.19 (0.06)^**^
Daily weight gain (g)	6.67 (13.15)	–
Intercept	–	76.56 (16.69)^***^

B = unstandardized beta, SE = standard error, Adjusted *R* square = 0.92 NPO = nil by mouth, DOL = day of life, GA = gestational age.

* *p* < 0.05,

** *p* < 0.01,

*** *p* < 0.001.

**Table 5.** Correlations (r2) between the feeding methods and three outcome variables.

**Variable**	**1**	**2**	**3**	**4**	**5**	**6**
1. LOH	1					
2. DOL to reach 2200g of BW	0.87^*^	1				
3. DOL when gavage feeding was started	0.36^*^	0.37^*^	1		0.40^*^	
4. DOL when nipple feed was started	0.88^*^	0.81^*^	0.38^*^	1	0.83	
5. DOL of full gavage & nipple feeds	0.83^*^	0.80^*^			1	
6. DOL of full nipple feeds	0.88^*^	0.86^*^	0.39^*^	0.84^*^	0.84^*^	1

LOH = length of hospitalization, DOL = day of life, BW = body weight,

* *p* < 0.001.

## Discussion

This study investigated the implications of bolus feeding given via oral or gastric routes on postnatal growth in very premature neonates. We examined the chronological age to achieve full enteral feeding, the minimum body weight corresponding to term status as the postnatal growth milestones and the duration of hospitalization. The results suggest that bolus feeding supplemented through an orogastric tube and bypassing oral suck and swallow function has no clinical contribution to these outcomes unless combined with nipple feeding, whereas nipple bottle feeding independently accelerates the achievements of total enteral nutrition and catch-up growth and reduces hospitalization duration in VPN. The start day of nipple feeding was found to be a strong determinant of the three tested postnatal outcome measures. The start date of BOG feeding, while having no independent associations, revealed a weak though highly significant relation with postnatal growth and discharge age of VPN, underscoring its small and interdependent role in their nutritional management. The postnatal maturation statuses were different for the two modalities at the start of feeding, being three to four days for orogastric and about two weeks for oral nipple feeding as clinically mandated. A Cochrane meta-analysis, which did not distinguish between continuous and bolus orogastric feeding methods, concluded that trophic orogastric feeding has no role in enhancing gut function, improving feeding tolerance, and reducing hospital stay in preterm infants [12, 13]. According to another meta-analysis, continuous OG feeding trends to take longer to achieve full feeding than bolus OG feeding [14]. Our study eliminated the potentially confounding effects of continuous OG feeding on the results by exclusively examining the bolus gastric feeding method. The results specified the limits and scope of the contribution of bolus orogastric feeding to the postnatal enteral nutrition management of prematurely born infants administered until they can feed orally.

Prior studies have reported inadequate enteral nutrition to be a barrier to discharge from the hospital in moderately preterm infants. Earlier introduction of oral feeding is demonstrated to accelerate the achievement of full feeding [11, 15]. The referred studies did not specify if the feedings were supplemented as only orogastric (OG) or as combined OG and oral or whether the OG feedings were provided as continuous, bolus or mixed methods. We examined the catch-up growth to term body weight as an indicator of postnatal growth for the first time and demonstrated that this process is enhanced by the acquisition of full enteral oral and combined gastric and oral feedings but not by bolus gastric feeding. Oral nipple feeding is physiological, unlike orogastric tube feeding, and is reported to induce local gastrointestinal hormones and contribute to the system’s functional and anatomical development [16]. Nonnutritive sucking is demonstrated to facilitate the transition from gavage to full oral feeding and reduce the duration of hospitalization [17]. Our results might indirectly highlight the beneficial effects of nutritive suck-and-swallow activities on postnatal growth, which are recruited during nipple feeding but bypassed by gastric bolus feeding. Our results have suggested that it may be safe to start nipple feeding at 32 weeks of post-menstrual age (PMA) in clinically stable VPN who have no significant apnea, bradycardia or desaturation at rest or during nonnutritive sucking, which is a week earlier than the currently practiced 33–34 weeks of PMA [11,18]. The introduction of nipple feeding at 32 weeks of post-menstrual age (PMA) [11,18] did not result in any significant adverse or untoward events. The reported fetal maturational age for the suck-swallow function is 33–34 weeks. Premature birth may enhance the timeline of developmental milestones and modify the trajectory of maturational processes in neonates compared to the fetus. Brumbaugh et al. introduced oral feeding at 33.9 weeks of postmenstrual age and demonstrated that the earlier start of oral feeds by one week reduces the time taken to achieve full feeding by 4–5 days [11]. The total number of infants born between 28–33 weeks of gestation in the year 2015 was 107,538 in the USA [19], and the average total cost of care was reported as $76,153 for infants born at <37 weeks of gestation and $114,437 for those who weighed <2500 g at birth [20]. If clinically permissible, deliberate initiation of nipple feeding at 32 weeks of postmenstrual age may be safe and successful in stable neonates and diminish their duration of hospitalization and cost of care.

We identified the intake of antibiotics as an independent risk factor for prolonged hospitalization in very preterm neonates. In their evaluation of over 14,000 infants, Ting et al. concluded that prolonged empirical use of antibiotics in preterm infants is associated with increased odds of the composite outcome of death, BPD, NEC, retinopathy of prematurity, hospital-acquired infection and neurological injury [21]. They did not evaluate LOH [21]. Neonatal morbidities, namely respiratory distress syndrome, patent ductus arteriosus, sepsis, necrotizing enterocolitis and bronchopulmonary dysplasia (BPD), are known to delay hospital discharge in VPN [12]. These illnesses have signs and symptoms common to sepsis and are often associated with infection, for which they receive antibiotics. Our results support identifying and implementing quality improvement measures to limit the use of antibiotics in managing neonatal illnesses and exercise antibiotics stewardship. The judicious use of antibiotics and improved feeding strategies could shorten the LOH in preterm neonates.

## Strengths and weaknesses

This is a single-center retrospective study, and the number of included infants is not large, although the statistical significance of the results suggests adequacy of power. We investigated exclusively the bolus orogastric feeding method and the postnatal catch-up to term as a growth variable, unlike past reports. The association of antibiotic use with prolonged hospitalization in very premature infants was not documented before. Our infants were fed via an orogastric tube; therefore, the results do not apply to the nasogastric feeding practice. A Cochran review reported no difference between nasogastric and orogastric gavage methods in the time taken to achieve full feeding [22, 23]. The results of our study demonstrate associations and do not ascribe to cause-and-effect relationships between feeding practices and the tested outcomes.

## Conclusions

Oral nipple feeding with bottle is independently associated with accelerated postnatal catch-up growth and shortened duration of hospitalization in very preterm infants. Bolus orogastric feeding does not demonstrate such associations unless combined with oral nipple feeding to provide enteral nutrition. The relations between bolus orogastric feeding and postnatal growth and hospitalization duration, although statistically highly significant, are weak and not translatable to independent clinical significance. Nipple feeding may be successfully introduced at 32 weeks of postmenstrual age under close watch in clinically stable very preterm neonates. The use of antibiotics is associated with prolonged hospitalization and should be carefully limited in these infants.

## Abbreviations

VPN: Very preterm neonates
N: nipple bottle feeding
BOG: Bolus orogastric tube feeding
LOH: length of hospitalization
FEN: day of life to attain full combined nipple and orogastric feeding
Wt22: bodyweight of 2200g
GA: gestational age
BW: birth weight
DOL: day of life
